The article "Probe into the Role of Music Therapy in Workplace Health Management" was retracted in 2023. Reasons: signs of a paper mill; suspected computer-generated content; unreliable results or conclusions; lack of ethics approval or compliance.

# Probe into the Role of Music Therapy in Workplace Health Management

**DOI:** 10.1155/2022/9999905

**Published:** 2022-03-04

**Authors:** Gang Li

**Affiliations:** Conservatory of Music Hanshan Normal University, Chaozhou 521041, Guangdong, China

## Abstract

With the rapid development of modern society, the rhythm of people's life and work is also forced to speed up. Stress from various fields makes people's health worse and worse. There are all kinds of pressures, and everyone in the torrent of the times has to face them. All kinds of pressures include life pressure, study pressure, and work pressure. Work pressure mainly comes from the pressure source, the individual's cognition of the pressure source, and the state of tension. Once too much work pressure is generated, it will bring unnecessary trouble to employees' lives and work and will also affect the company's interests. How to effectively alleviate work pressure is a problem that we urgently need to solve now. Specific problems are analyzed in detail. First, analyze the causes of work pressure. First, the pressure source is identified, and the pressure source generally exists objectively. It generally includes heavy work tasks, long working hours, and frequent job transfers. It is not easy to go through the employees themselves. Second is change, so this requires changing the individual's perception of the source of stress and the state of tension. In the continuous practice and research process of predecessors, some effective methods have been found, and music therapy is one of many methods, and music therapy has a wider range of effects and longer-lasting effects. This article mainly introduces how to effectively use music therapy in the work environment. It also includes a specific analysis of specific problems. The employees are mainly divided into mental workers and manual workers, and they are provided with different music therapy programs. The role of music therapy in workplace health management is such that it can effectively alleviate the work pressure of employees, enhance the feelings between employees, and improve the work efficiency of employees. Finally, the paper is summarized.

## 1. Introduction

With the rapid development of society, the pace of people's life and work has become faster and faster, which will cause people to face more and more pressure in their lives and work. At this stage, music therapy has been widely used, and many excellent results have been produced in the field of theoretical research [1]. Some scholars focus on the medical field, and some scholars apply it to adolescent psychological education [2]. All in all, regardless of the field, the positive significance of music therapy has been widely recognized.

The article "Probe into the Role of Music Therapy in Workplace Health Management" was retracted in 2023. Reasons: signs of a paper mill; suspected computer-generated content; unreliable results or conclusions; lack of ethics approval or compliance.

How to effectively alleviate the work pressure of employees in the workplace? This article summarizes some effective methods.

1. Sit and rest: relax, take a deep breath, and think of something pleasant.
2. Listening to music, good music can relax employees' moods and ease their tension
3. Talking like others can not only relieve pressure effectively, but also get new working ideas in the process of talking and communicating

Comparing these three methods, it can be found that the first and third methods take up a certain amount of time. It is impossible to achieve when you are busy at work, but the second method does not require time for music therapy. Even if you are busy at work, you can also work while listening to music [3], and music therapy has a wider coverage and longer duration of action. Therefore, this article mainly conducts related research on music therapy. In 1940, the United States made music therapy a complete and independent subject. Since then, the United States has always occupied a leading position in the development of modern music therapy in the world [4]. The earliest music therapy in China appeared in “The Yellow Emperor's Classic of Internal Medicine.” China's modern music therapy began in the 1980s and has a history of more than 40 years. Music therapy in China has formed a preliminary and relatively complete theory and application system.

## 2. Effective Use of Music Therapy in the Work Environment

### 2.1. Work Pressure and Music Therapy

Work pressure is a dynamic situation. Effectively alleviating work pressure requires the right remedy for these factors [2]. The source of stress exists objectively and is not easy to change through external forces. Therefore, it is necessary to address the factors of an individual's perception of the source of stress and the state of tension.

Music therapy refers to the use of music to regulate the physiology and psychology of living organisms. The physical energy generated by musical works to stimulate the development and transformation of human cells in the desired direction. There are various methods of music therapy, which can be divided into receptive, improvised, and recreative. The main types of acceptance include music listening and music discussion. Recreation requires a certain degree of creative ability, and some new related creations need to be produced, which are mainly divided into psychological musical drama, song creation, or music composition. Impromptu music, as the name suggests, is improvisation, such as whistling, verbal improvisation, and instrument improvisation.

### 2.2. Work Environment

In the actual work environment, the receptive method can be realized by installing a radio in the work environment. Employees can listen to songs through the radio. For workers who are mainly engaged in mental labor at work in the company, the content of the songs can be light music. The more cheerful music can inspire the creativity of employees, sounds comfortable, and can relieve fatigue. It is best not to be rock or heavy metal or even darker music. This music may have a counterproductive effect and cause employees to feel bad emotions. The time period for playing music can be the start time in the morning, the end time of the nap, and the overtime in the evening. It is best to play music for about five to ten minutes; otherwise, it may cause aesthetic fatigue to employees. It is best to change the played songs in three to five days. It is not possible to listen to only one song for a long time, which will also cause the aesthetic fatigue of employees and lose the effect of music therapy [5]. For workers who are mainly engaged in assembly line manual labor at the factory, it is best to play music that is preferred by the employees. The sound of the music can be louder because there are more noises in the factory, and the louder music can be properly concealed. The time period for playing music can be most of the working hours. The length of playing music can be adjusted with working hours. It is best to change the cycle of playing songs in two to three days, and it is also not possible to listen to only one song for a long time. Music discussion can be realized by creating a music exchange meeting. Employees can join the exchange meeting to exchange their music experiences after work, or share the work environment music broadcasting platform, where employees can provide some suggestions for playing music.

The article "Probe into the Role of Music Therapy in Workplace Health Management" was retracted in 2023. Reasons: signs of a paper mill; suspected computer-generated content; unreliable results or conclusions; lack of ethics approval or compliance.

The recreative method can be realized by holding internal competitions or related music activities. After work, the company can carry out some related competitions or activities such as singing, composing, and writing lyrics to mobilize the enthusiasm of employees and relieve employees' enthusiasm [6].

The improvisational music method can be realized by carrying out a music tea party or a dinner party. During the meeting or during the dinner party, employees can improvise their talents, which can show themselves and enliven the atmosphere.

This concludes a diagram of the effective use of music therapy in the work environment, as shown in Figure 1.

The effective use of music therapy in the work environment has played a positive role in workplace health management. It can not only effectively relieve the work pressure of employees and reduce the psychological burden of employees at work, but also shorten the distance between employees and increase the distance between employees. The feelings of the company can improve the cohesion and centripetal force of the company, and it can also mobilize the enthusiasm of employees, greatly improve the work efficiency of employees, and bring greater benefits to the company.

## 3. Relieve Employees' Stress

### 3.1. Receptive Methods

Using receptive methods to play music for employees through radio or other channels can effectively alleviate employee pressure [7]. Listening to music can affect the emotional state of employees, and it can change employees' perception of time and space at work, just as one person might devote themselves wholeheartedly to doing a happy thing and feel that time passes quickly. When they are doing something that they do not like, they will become anxious, feel that time is passing slowly, passing the day like a year, and wonder if time can be any faster, and every second feels like a kind of suffering. Listening to music can also relieve physiological changes, reduce anxiety and stress, and make employees feel relaxed. The specific operation method is shown in the figure.

### 3.2. Work Type Experiment

The work types are mainly divided into company employees engaged in mental work and factory employees engaged in manual labor. For company employees engaged in mental work, the morning hours are the best time of the day to work. The morning is the beginning of a good day. Whether having a good mood in the morning is crucial to the smoothness of the day's work. Therefore, it is very important to play appropriate music for company employees five to ten minutes after the start of work in the morning. Healthy and gentle music can not only promote the metabolism of the body's internal organs and relieve muscle fatigue, but it can also provide employees with psychological comfort, give them a mental massage, let them put aside the distracting thoughts in their minds and the pressure in their hearts, and devote themselves to the day's work. When it is a hot day after the employee's lunch break, at this time, employees' hearts are usually more impetuous and hot. This requires cool medicine to reduce the fire. Fresh and cool light music may be very suitable for this time. Employees with impetuous hearts can effectively alleviate their irritable moods. If you need to work overtime at night, the employees' bodies must be very tired at this time, and they may be anxious to go home, and their hearts will be restless. At this time, a warm, loving, and motivating song is undoubtedly for them. Sending charcoal into the snow can help relieve their physical and physical fatigue. For factory employees engaged in manual labor, they may need to work on an assembly line for more than ten hours and sometimes even need to stay up late. With boring and boring work coupled with long-term uninterrupted repetition of the already harsh machine noise, it makes employees feel stressed and anxious and reduces their motivation at work. Therefore, it is necessary to introduce the music they like to employees to cover the noise that makes them anxious and to relieve their work pressure to a certain extent. Fast-paced music can make employees' emotions more elevated, enhancing the employees' passion for work; slow-paced music can effectively relieve muscle fatigue, calm the employees' hearts, and achieve a combination of work and rest. Carrying out a music exchange meeting can also alleviate the pressure of employees. Try to arrange the time of the exhibition and exchange meeting on a relatively idle working day. Do not occupy the employees' personal rest time. Taking up the employees' rest time will make the employees disgusted. The effect can only be that it is counterproductive. Carrying out similar music activities can make employees temporarily forget the troubles and pressures at work. When they devote themselves to it, they can relax physically and mentally and enjoy their work better. More fun from work. Carrying out singing, word-making competitions or activities, and holding camellia parties and dinner parties can also make employees feel relaxed, cultivate sentiment, and let them feel the joy of work [8]. As a result, a survey was conducted. The purpose of the survey is to understand whether these activities can relieve the work pressure of employees. The subjects of the survey are 50 company employees engaged in mental work and 50 factory employees engaged in physical activities. The male-to-female ratio is 1:1. The age range is 23 to 45 years old, and the survey results obtained are shown in Table 1.

The article "Probe into the Role of Music Therapy in Workplace Health Management" was retracted in 2023. Reasons: signs of a paper mill; suspected computer-generated content; unreliable results or conclusions; lack of ethics approval or compliance.

From this questionnaire, we can see that company employees engaged in mental work and factory employees engaged in manual labor are more inclined to broadcast. The approval rates are as high as 96% and 92%. However, it can be clearly observed that these employees are the ones who are in need of activities to relieve work pressure. It has relatively the lowest approval rate, but even the lowest approval rate is 62%, more than half. Therefore, practice shows that the use of music therapy can indeed effectively relieve the work pressure of employees.

## 4. Enhance Employee's Feelings

### 4.1. Forms of Enhance Employee's Feelings

Music therapy can not only effectively alleviate the work pressure of employees but also enhance the feelings between employees. First of all, because music therapy can relax the mood of employees and make their physical and mental states more content. This is not only conducive to effective communication between employees, but also can arouse the emotions of employees wanting to understand each other and enhance friendship, and this kind of good effective communication can also create a harmonious atmosphere and form a virtuous circle, which can not only delight the mood of employees but also enhance the cohesion and centripetal force of the working environment [9]. People who are full of stress and in a bad mood are self-enclosed and even hurt others with bad words. Only those who are in a good mood will think about communicating with others, and in the process of communicating, they can still infect each other so that they can pass on happiness and form a positive, friendly, and mutually helpful atmosphere. Secondly, music therapy can provide employees with various channels to understand and communicate with each other. Whether it is participating in music exchange meetings, competitions, or other activities such as camellia parties and dinners, employees can build a platform for mutual understanding and communication. They are mutual help partners at work, close friends in life, and even harvest love in these music-related activities, and also find like-minded partners at work who also like music. After work, you can meet to sing, listen to concerts, and watch musicals. Music is a bridge between people's hearts, and music therapy opens a window between employees at work. A survey was also carried out.

### 4.2. Summary of Experimental Data

The purpose of the survey was to find out whether these activities can enhance the working feelings of employees. The subjects of the survey were 50 company employees engaged in mental work and 50 factory employees engaged in physical activities. The ratio of male-to-female was 1 : 1. The age range was 23 to 45 years old. The survey results obtained are shown in Table 2.

From this questionnaire, we can see that company employees engaged in mental work and factory employees engaged in manual labor are more inclined to the way of camellia parties or gatherings, and the approval rate is as high as 94% and 84%, respectively, found from comparing the forms of camellia parties or gatherings. It is direct and does not take up too much rest time, so employees are more inclined to enhance their friendship with each other in this way. The broadcast method lacks interaction between employees, so the approval rate is the lowest, at only 52%, but it is more than half. In short, the way to report competitions or some activities or dinner parties can effectively enhance the relationship between employees.

The article "Probe into the Role of Music Therapy in Workplace Health Management" was retracted in 2023. Reasons: signs of a paper mill; suspected computer-generated content; unreliable results or conclusions; lack of ethics approval or compliance.

## 5. Improve Employee Work Efficiency

### 5.1. Positive Significance in Improving Work Efficiency

Music therapy can not only effectively alleviate the work pressure of employees and enhance the feelings between employees, but also improve the work efficiency of employees [10, 11]. Work efficiency depends on the work status of the employees and the collaboration between employees or departments [12, 13]. The working status of employees depends on their working environment, their physical energy, and their mental spirit. Music therapy can provide employees with a good and comfortable working environment and a friendly and mutually helpful working atmosphere. It can effectively relieve the physical and mental pressure of employees so that they are no longer exhausted but full of motivation and can provide employees with plenty of energy and full spirit [14, 15]. Having such a good working condition can naturally improve the work efficiency of employees. Because music therapy is conducive to enhancing the feelings between employees, it will make the linkage and cooperation between employees or departments more tacit[16]. A more tacit and faster linkage and cooperation between employees or departments can naturally greatly improve the work efficiency of employees [17, 18]. It can also save more costs for the company, bring greater benefits, seek more benefits for the employees themselves, and form a virtuous circle. It can make every employee feel a sense of belonging and accomplishment and enhance their happiness in the company. As a result, a survey was conducted.

### 5.2. Summary of Experimental Data

The purpose of the survey is to understand whether these activities can improve the efficiency of employees [19, 20]. The subjects of the survey are 50 company employees engaged in mental work and 50 factory employees engaged in physical activities. The male-to-female ratio is 1:1. The age range is 23 to 45 years old, and the survey results obtained are shown in Table 3.

From this questionnaire, we can see that company employees engaged in mental work and factory employees engaged in manual labor are more inclined to broadcast, and the approval rate is as high as 98% and 96% because the broadcast method has a wider coverage and employees are more involved, and it is the only one that can be passively accepted. In addition, employees are more inclined to the way of camellia parties or gatherings, with approval rates reaching 88% and 90%, respectively. At the same time, it can be clearly observed that these employees have the lowest approval rate for using competitions or activities to improve their work efficiency, but even the lowest approval rate is 70%, more than half. So practice shows that the use of music therapy can indeed effectively improve employee work efficiency.

The article "Probe into the Role of Music Therapy in Workplace Health Management" was retracted in 2023. Reasons: signs of a paper mill; suspected computer-generated content; unreliable results or conclusions; lack of ethics approval or compliance.

## 6. Conclusion

Reasonable use of music therapy can effectively alleviate employees' stress, improve employees' moods, and energize employees. It is also conducive to the consolidation of employee relationships, enhances the relationship between employees, strengthens the connection between each department, and enhances employees' sense of belonging and happiness, all of which help to improve the work efficiency of employees, increase the company's profits, and form a virtuous circle.

According to the survey, employees generally believe that the broadcasting method is very conducive to directly alleviating work pressure and improving work efficiency. Therefore, we can write more articles on the broadcasting method in music therapy and increase the interaction between employees. In terms of enhancing employee feelings, employees generally agree with the way of tea chat or gathering, because this method does not take up the employees' private rest time too much and the time is generally not too long. It is not easy to disgust employees, and employees are also willing to actively participate in it. Passive acceptance and active participation are combined to maximize the role of music therapy in workplace health management. In future research, the specific effects of the application of different music types in the work environment will be focused on to find out the most suitable music types for health management in various industries.

## Figures and Tables

**Figure 1:** Realization diagram of music therapy in working environment.

**Table 1:** Questionnaire on the effect of music therapy on relieving work pressure.

	Number	Can broadcasting relieve work pressure?			Whether the music exchange meeting can relieve work pressure			Whether competitions or activities can relieve work pressure				Can a camellia party or a dinner party alleviate work pressure?			
		Yes	No	Approval rate (%)	Yes	No	Approval rate (%)	Yes	No	Approval rate (%)	Yes	No	Approval rate (%)
Mental worker	50	48	2	96	42	8	84	40	10	80	43	7	86

Physical worker	50	46	4	92	38	12	76	31	19	62	40	10	80

**Table 2:** Questionnaire on the effect of music therapy on enhancing employees' feelings.

	Number	Can broadcasting enhance the feelings of employees?			Whether the music exchange can enhance the feelings of employees			Whether competitions or activities can enhance the feelings of employees			Whether the camellia party or dinner can increase the feelings of the employees (improvisation)?		
		Yes	No	Approval rate (%)	Yes	No	Approval rate (%)	Yes	No	Approval rate (%)	Yes	No	Approval rate (%)
Mental worker	50	30	20	60	46	4	92	45	5	90	47	3	94

Physical worker	50	26	24	52	41	9	82	38	12	76	42	8	84

The article "Probe into the Role of Music Therapy in Workplace Health Management" was retracted in 2023. Reasons: signs of a paper mill; suspected computer-generated content; unreliable results or conclusions; lack of ethics approval or compliance.

**Table 3:** Questionnaire on music therapy for improving employees' work efficiency.

	Number	Can broadcasting be able to improve the work efficiency of employees?			Whether the music exchange meeting can improve the work efficiency of employees			Whether competitions or activities can improve employee productivity			Can a camellia party or a dinner party improve the work efficiency of employees?		
		Yes	No	Approval rate (%)	Yes	No	Approval rate (%)	Yes	No	Approval rate (%)	Yes	No	Approval rate (%)
Mental worker	50	49	1	98	41	9	82	39	11	78	44	6	88

Physical worker	50	48	4	96	37	13	74	35	15	70	45	5	90

## Data Availability

The datasets used and/or analyzed during the current study are available from the corresponding author on reasonable request.
